RETRACTED

# Huayu Tongluo Recipe Attenuates Renal Oxidative Stress and Inflammation through the Activation of AMPK/Nrf2 Signaling Pathway in Streptozotocin- (STZ-) Induced Diabetic Rats

**DOI:** 10.1155/2021/5873007

**Published:** 2021-07-28

**Authors:** Yachun Li, Shuai Guo, Fan Yang, Lifei Liu, Zhiqiang Chen

**Affiliations:** ^1^Hebei University of Chinese Medicine, Shijiazhuang 050091, China; ^2^Hebei Hospital of Traditional Chinese Medicine, Shijiazhuang 050091, China

## Abstract

Diabetic nephropathy (DN), a severe microvascular complication of diabetes, is one of the leading causes of end-stage renal disease. Huayu Tongluo Recipe (HTR) has been widely used in the clinical treatment of DN in China, and its efficacy is reliable. This study aimed to explore the renoprotective effect of HTR and the underlying mechanism. Male Sprague-Dawley rats were fed with high sugar and fat diet combined with an intraperitoneal injection of STZ to establish the diabetic model. Rats in each group were respectively given drinking water, HTR, and irbesartan by gavage for 16 weeks. 24-hour urine samples were collected every 4 weeks to detect the content of total protein and 8-OHdG. Blood samples were taken to detect biochemical indicators and inflammatory markers at the end of 16th week. Renal tissue was collected to investigate pathological changes and to detect oxidative stress and inflammatory markers. AMPK/Nrf2 signaling pathway and fibrosis-related proteins were detected by immunohistochemistry, immunofluorescence, real-time PCR, and western blot. 24h urine total protein (24h UTP), serum creatinine (Scr), blood urea nitrogen (BUN), total cholesterol (TC), and triglyceride (TG) were decreased in the rats treated with HTR, while there was no noticeable change of blood glucose. HTR administration decreased malondialdehyde (MDA) content and increased superoxide dismutase (SOD) activity in kidneys, complying with reduced 8-OHdG in the urine. The levels of TNF-*α*, IL-1*β*, and MCP1 and the expression of nuclear NF*κ*B were also lower after HTR treatment. Furthermore, HTR alleviated pathological renal injury and reduced the accumulation of extracellular matrix (ECM). Besides, HTR enhanced the AMPK/Nrf2 signaling and increased the expression of HO-1 while it inhibited the Nox4/TGF-*β*1 signaling in the kidneys of STZ-induced diabetic rats. HTR can inhibit renal oxidative stress and inflammation to reduce ECM accumulation and protect the kidney through activating the AMPK/Nrf2 signaling pathway in DN.

## 1. Introduction

Diabetic nephropathy (DN), with high mortality and disability rate, is one of the most severe microvascular complications and has become the leading cause of the end-stage renal disease (ESRD) in most countries [1]. As a primary treatment approach, strict glycemic and blood pressure control is not only challenging to maintain, but also cannot prevent DN from developing ESRD. Therefore, prevention and treatment of DN is becoming increasingly urgent.

RETRACTED

The primary clinical manifestation of DN is mass proteinuria. Moreover, the key pathological change is the proliferation of extracellular matrix (ECM), which leads to the thickening of the glomerular basement membrane (GBM) and finally develops glomerulosclerosis [2]. Transforming growth factor *β*1 (TGF-*β*1) is a well-known fibrogenic factor, which can promote the production of ECM protein and reduce its degradation at the same time. Oxidative stress, caused by excessive production of reactive oxygen species (ROS), plays a vital role in the pathogenesis of DN. And it is the main reason for the high expression of TGF-*β*1 in the kidney [3, 4]. Furthermore, NADPH oxidase (Nox) has emerged as a major source of ROS in DN. Also, the high expression of Nox4 directly upregulates TGF-*β*1 signaling via TGF-*β* receptor Ι, leading to diabetic kidney hypertrophy and the accumulation of ECM, including fibronectin (FN) and type IV collagen (Col IV) [5, 6].

In addition to oxidative stress, the role of inflammation in DN has also received extensive attention. Inflammation is considered to predict the process of DN and persistent microalbuminuria in patients with type 2 diabetes, independently of traditional risk factors [7]. The events in diabetes, such as hyperglycemia and advanced glycation end products (AGEs), upregulate the expression of NF*κ*B (the proinflammatory transcription factor), resulting in the infiltration of inflammatory cells in the diabetic kidney, which secrete proinflammatory cytokines and ROS, facilitating the development of fibrosis in DN [8, 9]. Furthermore, oxidative stress and inflammation can interact with each other for positive feedback regulation and aggravate the kidney damage of DN [10, 11]. However, compared with the proinflammatory pathways, our understanding of anti-inflammatory pathways is insufficient [12]. 5′Adenosine monophosphate-activated protein kinase (AMPK) is well known as an energy sensor in cells, which can regulate glucose and lipid metabolism and maintain the balance of energy metabolism [13]. In recent years, it has been shown that AMPK, abundantly expressed in the kidney, is also the main intracellular ROS sensor [14]. Moreover, it has obvious antioxidant [15] and anti-inflammatory [16] effects in the kidney cells, which have been reported to be related to nuclear factor E2-related factor 2 (Nrf2) pathway partly [17, 18]. AMPK acts on the upstream of the Nrf2-antioxidant response element (ARE) pathway [19], which plays a key role in the antioxidant defense mechanism. When the Nrf2 pathway is activated, it is released into the nucleus, which is followed by binding to the ARE sequence of downstream target genes (NADPH quinone oxidoreductase-1 [NQO-1], heme oxygenase-1 [HO-1], and glutathione S-transferase [GST]) to neutralize free radicals and accelerate the clearance of cytotoxin [20]. In addition, Nrf2 can activate antioxidant cascades to combat inflammation [21]. Therefore, it is also considered to be an anti-inflammatory pathway. Taken together, we consider that the AMPK/Nrf2 signaling pathway is closely related to renal inflammation and oxidative stress in DN. How to improve the activity of AMPK/Nrf2 signaling and whether it can alleviate kidney injury has become a focus of our research.

RETRACTED

In recent years, natural medicine, including traditional Chinese medicine (TCM), has been extensively studied and applied in chronic kidney disease. Huayu Tongluo Recipe (HTR) is a compound prescription composed of *Salvia miltiorrhiza* Bge., Rhizoma Ligustici Wallichii, *Pheretima aspergillum*, *Aulastomum gulo*, and Scorpio, aiming to ‘promote blood circulation and resolve stasis' and ‘dredge collaterals.' It is widely used in the prevention and treatment of DN and has a reliable efficacy. Our previous studies have confirmed that HTR can effectively reduce urinary protein excretion and improve renal fibrosis in diabetic rats [22]. Many pharmacological studies have shown that the active ingredients included in HTR have antioxidant and anti-inflammatory effects to delay fibrosis [23, 24]. In summary, we have sufficient reasons to hypothesize that HTR protects the kidney against oxidative stress and inflammation via the AMPK/Nrf2 signaling pathway in DN, thereby inhibiting renal fibrosis and reducing urine protein.

## 2. Methods

### 2.1. Drugs

HTR is composed of Radix Salviae Miltiorrhizae (15g), Rhizoma Ligustici Wallichii (12g), *Pheretima aspergillum* (10g), *Aulastomum gulo* (6g), and Scorpio (6g). All the components were donated in the form of formula granules by Guangdong Yifang Pharmaceutical Co., Ltd. (Foshan, China). Irbesartan dispersion tablet was purchased from China Resources Double-Carne Pharmaceutical Co., Ltd. (Jinan, China).

### 2.2. Drugs

Healthy male 4-week-old Sprague-Dawley (SD) rats weighing about 60–80 g were purchased from Beijing Vital River Laboratory Animal Technology Co., Ltd. The rats were housed in a standard environment room with temperature 24 ± 1°C, illumination (12h light/12h dark cycles), and relative humidity of 50%–70%. The study was approved by the Ethics Committee of Hebei Provincial Hospital of Traditional Chinese Medicine and carried out in accordance with Guidance Suggestions for the Care and Use of Laboratory Animals published by the Ministry of Science and Technology of China.

RETRACTED

### 2.3. Animal Modeling and Grouping

After 1 week of acclimatization, all rats were randomly separated into control group (*n* = 7) fed with common food (3.51 kcal/g) and model preparing group (*n* = 33) fed with high-fat diet (4.43 kcal/g). After six weeks, the rats in the model preparing group were intraperitoneally injected with STZ 35 mg/kg (diluted with 0.1 M pH 4.3 sodium citrate solution to 1%). The blood glucose was measured after 72 hours. The blood glucose ≥16.7 mM is the criterion for successful diabetes model. 2 rats did not meet the modeling standards and were eliminated, and 3 rats died within 72 hours after STZ injection. The rest of the rats were randomly divided into model group (*n* = 10), HTR treatment group given HTR (4.59 g/kg daily by gavage, *n* = 9), and irbesartan group given irbesartan dispersion tablet (13.5 mg/kg daily by gavage, *n* = 9). Furthermore, the rats in the control and model groups were gavaged with an equal volume of drinking water. The random blood glucose was measured every 4 weeks with an ACCU-CHEK® Performa glucometer (Roche, Hoffmann, Germany), and those with blood glucose <16.7 mM were eliminated. During the 16-week research period, 3 rats in the model group, 2 rats in the irbesartan group, and 2 rats in the HTR group died. After 16 weeks of gavage, the remaining rats were euthanized. And the samples of blood, urine, and kidneys were collected to detect the parameters.

### 2.4. Biochemical Parameters

The rats' urine was collected for 24 hours on the 1st day and the end of 4th, 8th, 12th, and 16th week after gavage to detect the 24h UTP excretion. Blood in vacuum tubes was centrifuged at 3500 rpm for 15 minutes, and the serum was taken to detect the renal function (Scr and BUN) and blood lipids (TC and TG) by an automatic biochemical analyzer (Hitachi, Japan). MDA, SOD, interleukin-1*β* (IL-1*β*), tumor necrosis factor-*α* (TNF-*α*), and monocyte chemoattractant protein-1 (MCP-1) were tested using commercially available kits (JianCheng Bioengineering Institute, Nanjing, China).

### 2.5. Renal Morphologic Analysis

One-third of kidneys were fixed with 4% paraformaldehyde for 48h, and then these tissues were sliced into approximately 2 *µ*m sections and stained by hematoxylin-eosin (HE), periodic acid-Schiff (PAS), and Masson's trichrome. The kidney morphology was observed, and the images were acquired by a light microscope (Olympus, Japan).

### 2.6. Immunohistochemical (IHC) and Immunofluorescence (IF) Staining

Paraffin-embedded kidney tissue was sectioned into 2 µm thickness. Sections were deparaffinized in xylene and then rehydrated in graded reducing ethanol concentrations (100%, 95%, 80%, 70%, and 50%, respectively). The sections were put into the repair solution and repaired with high pressure for 5 min. Moreover, endogenous peroxidases were diminished using 3% hydrogen peroxide for 10 min. The sections, which were conducted by IHC, were blocked with goat serum and incubated with primary antibodies (FN, 1 : 200, Abcam, USA, 89443; Col IV, 1 : 200, 6586, and 8-OHdG, 1 : 200, Japan Institute for the Control of Aging, Japan, MOG-020P) overnight at 4 °C. Then biotinylated goat secondary antibody and streptavidin-HRP were dropped onto slides in turn. Diaminobenzidine (DAB) was used for the color reaction, which was followed by counterstaining with hematoxylin. The sections, which were conducted by IF, were blocked with nonspecific epitopes with 5% BSA and then immunoassayed with primary antibodies (Nrf2, 1 : 100, Bioss, China) overnight at 4°C. DAPI staining solution was used to stain cell nucleus. At last, all slices were mounted with gummy neutral balsam.

RETRACTED

### 2.7. Real-Time Quantitative Polymerase Chain Reaction (qRT-PCR)

Total RNA of the renal cortex was extracted with the TRIzol Reagent (Servicebio, Wuhan, China). The purity and concentrations were tested by a NanoDrop2000 spectrophotometer (Thermo Scientific, Waltham, USA). Then the RT First Strand cDNA Synthesis Kit (Servicebio, Wuhan, China) was used to reverse-transcribe the RNA into cDNA. The primers of each gene (shown in Table 1) were designed by Primer 5.0 and synthesized by Servicebio (Wuhan, China). The PCR was carried out using 2×SYBR Green qPCR Master Mix (Servicebio, Wuhan, China) on Fluorescence quantitative PCR instrument (ABI, USA). Each reaction was performed in triplicate. Taking GAPDH mRNA expression as a reference, levels of relative mRNA expression were calculated by the 2^−ΔΔCt^.

### 2.8. Western Blot

The frozen kidney tissue was homogenized in RIPA buffer (BestBio, Shanghai, China), and the protein content was determined by the BCA method. Equal amounts of protein were separated on 10% SDS-PAGE. The proteins were then transferred onto the PVDF membrane and were blocked using 5% skimmed milk. The membranes were incubated with primary antibodies all night at 4°C and then with secondary antibodies at room temperature. The enhanced chemiluminescence (ECL) detection (Millipore, MA, USA) was utilized to make the membranes visualized. At last, the destination band was scanned and quantified using the infrared fluorescence imaging system (Odyssey, USA).

RETRACTED

The primary antibodies used in this study are as follows: AMPK*α* (1 : 800, Cell Signaling Technology, USA, 5831), p-AMPK*α* (1 : 1000, 2535), Nrf2 (1 : 1000, Abcam, USA, 89443), Nox4 (1 : 1000, 133303), TGF-*β*1 (1 : 600, 215715), HO-1 (1 : 1000, Santa Cruz, USA, 390991), NQO1 (1 : 1000, 376023), and NF*κ*B (1 : 600, Servicebio, China, 11997).

### 2.9. Statistical Analysis

All data are presented as mean ± standard deviation. Comparison between groups was performed by one-way ANOVA with LSD-t's multiple comparisons using SPSS 25.0 software (IBM, NY, USA). *P* value <0.05 was regarded as a statistically significant difference.

## 3. Results

### 3.1. Effects of HTR on 24h UTP and Renal Function

As presented in Figure 1(a), after 4, 8, 12, and 16 weeks of intervention, the 24h UTP of the model group was increased significantly compared with the control group. Treatment with HTR and irbesartan significantly decreased 24h UTP, and there was no statistical difference between the two treatment groups. BUN (Figure 1(b)) and Scr (Figure 1(c)) in the model group were significantly higher than those in the control group. HTR and irbesartan administration remarkably reduced Scr and BUN, and there was no statistical difference between the two treatment groups.

### 3.2. Effects of HTR on Random Blood Glucose (RBG) and Blood Lipids

The RBG (Figure 2(a)) of all rats was higher than that of the control group in the experimental period of 16 weeks, and the intervention with HTR and irbesartan did not reverse the RBG. However, as illustrated in Figure 2(b), HTR did reduce the TC and TG significantly.

### 3.3. Effects of HTR on the Renal Pathology of STZ-Induced Diabetic Rats

HE, PAS, and Masson's trichrome were used to investigate the histopathological changes of kidneys. As shown in Figure 3, the renal structure was normal and clear in the control group. However, glomerular hypertrophy, noticeable thickening of the GBM, severe hyperplasia of mesangial cells, and significant accumulation of ECM were found in the kidneys of rats in the DN group. In contrast, treatment with HTR and irbesartan did alleviate the pathological renal injury of rats to varying degrees.

### 3.4. Effects of HTR on the Parameters of Oxidative Stress in Urine and Kidney

The activity of antioxidant enzyme SOD and the content of lipid peroxidation product MDA were jointly tested to reflect the degree of oxidative stress in kidneys. The SOD activity (Figure 4(a)) was decreased, and the MDA content (Figure 4(b)) was increased in the kidney tissue of rats in the model group. The SOD activity was higher, and the MDA content was lower in the two treatment groups than the model group. In addition, there was no statistical difference in the SOD activities between the two treatment groups. However, the effect of HTR on the reduction of MDA content was better than irbesartan.

8-Hydroxydeoxyguanosine (8-OHdG), an oxidized purine residue of DNA, has been recognized as an excellent marker of oxidative damage in tissue [25]. Thus levels of 8-OHdG in urine and kidney tissue were measured to assess the extent of the kidneys' oxidative damage. As presented in Figure 4(c), the urinary 8-OHdG level was amplified in the model group, and it was declined in the treatment groups. Immunohistochemical staining of 8-OHdG (Figure 4(d)) also presented the same result as the urine test. 8-OHdG is mainly located in the nucleus. The nuclear expression of 8-OHdG was higher in the DN rats' kidneys than that in the control group. And it was reduced after treatment with HTR and irbesartan.

RETRACTED

### 3.5. Effects of HTR on the Parameters of Inflammation in Serum and Kidney

TNF-*α*, IL-1*β*, and MCP1 in serum and mRNA expression in kidneys were tested to evaluate the extent of inflammatory response. In addition, the NF*κ*B expression in the kidney was also detected. As illustrated in Figure 5(a) and Figure 5(b), TNF-*α*, IL-1*β*, and MCP1 were significantly increased in the model group compared with the control group. The IL-1*β* level in serum (Figure 5(a)) and MCP1 mRNA expression (Figure 5(b)) were attenuated by irbesartan treatment. Moreover, HTR treatment could significantly reduce the levels of these inflammatory indicators in serum and the mRNA expression in the kidney (Figures 5(a) and 5(b)). In terms of NF*κ*B expression (Figures 5(c) and 5(d)), the total NF*κ*B in the model group was increased. And it was not reduced in the HTR and irbesartan group. However, HTR and irbesartan treatment markedly suppressed the nuclear translocation of NFkB, thereby inhibiting its activity. These results demonstrated that HTR could improve the inflammatory response of DN.

### 3.6. Effects of HTR on Nox4/TGF-*β*1 Signaling Pathway and the ECM Proteins

To understand the antifibrosis effect of HTR, western blot was used to detect the expression of Nox4/TGF-*β*1 signaling pathway, and immunohistochemistry was used to detect the expression of ECM proteins. The results revealed that the expression of Nox4 and TGF-*β*1 (Figures 6(a)–6(c)) was amplified considerably in the model group, complying with the increased expression of FN and Col IV (Figure 6(d)). Both HTR and irbesartan treatment inhibited the Nox4/TGF-*β*1 signaling pathway and restored the expression of FN and Col IV.

### 3.7. Effects of HTR on AMPK/Nrf2 Signaling Pathway

Real-time PCR (Figures 7(g) and 7(h)), western blot (Figures 7(a)–7(f)), and immunofluorescence were used to detect the activity of AMPK/Nrf2 pathway. The results showed that the phosphorylation of AMPK was significantly suppressed in the model group, and the total and nuclear Nrf2 expressions were decreased. Meanwhile, the mRNA and protein expressions of HO-1 and NQO1 were also declined. Irbesartan treatment only increased the pAMPK but had no significant effect on the other proteins in the pathway. HTR treatment stimulated the phosphorylation of AMPK and increased the nuclear translocation of Nrf2, although it cannot increase the expression of total Nrf2 compared with the model group. At the same time, the mRNA and protein expression of HO-1 were restored in the HTR group, although the NQO1 levels of mRNA and protein were not improved. Consistently with Nrf2 expression detected by western blot, immunofluorescence (Figure 7(i)) also revealed lower expression of nuclear Nrf2 in the model group and increased nuclear translocation of Nrf2 in HTR group. Therefore, we consider that HTR can reverse AMPK/Nrf2 activity in DN.

RETRACTED

## 4. Discussion

TCM is a discipline with a history of more than two thousand years. Overall concepts and dialectical treatment are the core of TCM theoretical system, derived from long-term clinical practice. It emphasizes the integrity of the body and its interrelationship with the natural and social environment. It is also considered that the treatment of disease is changing with the main symptoms and the stage of the disease. It has been reported that TCM has great advantages in the treatment of DN [26, 27]. However, because of its complex composition and lack of mechanism research, the application and development of TCM are limited. It is expected that this study can provide experimental evidence for the clinical application of HTR in the treatment of DN.

In this study, STZ-induced diabetic rats showed increased 24h UTP, upregulated Scr and BUN, complying with glomerular hypertrophy, thickened GBM, and increased ECM, which indicated that the diabetic rats developed DN. The main pathological manifestation of DN is the proliferation of ECM. And the massive accumulation of ECM results in renal fibrosis, eventually leading to renal failure and ESRD. This study showed increased collagen area and upregulated expression of FN and Col IV in kidney tissues of STZ-induced diabetic rats, both of which were significantly improved by HTR treatment. Therefore, we further studied its mechanisms. Oxidative stress and inflammation are considered to play a key role in TGF-*β*1-induced proliferation of ECM [28, 29]. Interestingly, there is a close relationship between oxidative stress and inflammation, which can accelerate the progression of DN [11]. ROS directly or indirectly activates NF*κ*B (the master regulator of innate and acquired immunity response) to stimulate the recruitment of inflammatory cells and the production of inflammatory cytokines involved in DN progression [30, 31]. In turn, the accumulation of cellular proinflammatory molecules (e.g., TNF-*α*) increases the generation of oxygen radicals and aggravates oxidative stress [32]. Therefore, we simultaneously detected indicators of oxidative stress and inflammation in STZ-induced diabetic rats.

RETRACTED

MDA is the final breakdown product of lipid peroxidation, and SOD is an enzyme of antioxidant defense system. 8-OHdG is a marker of DNA oxidative damage. When excessive ROS cannot be eliminated by the antioxidant defense system, it can trigger oxidative stress. Increased content of MDA, decreased activity of SOD, and increased excretion and expression of 8-OHdG are all signs of oxidative stress in the body, which appeared in the results of this research. As we all know, one of the main sources of ROS in the kidney is derived from NADPH oxidase [33]. Nox4, a subtype of NADPH oxidase, is abundantly expressed in the kidney. And its expression is significantly increased in DN. Researchers suggested that Nox4-sensitive pathways mediate the enhanced TGF-*β*1 and FN levels to promote the process of renal fibrosis in type 2 DN [34]. Therefore, we, meanwhile, detected the activity of Nox4/TGF-*β*1 signaling pathway. Together with the above indicators, it reflects the degree of oxidative stress. Our data showed that the activity of Nox4/TGF-*β*1 signaling pathway was intensified in the STZ-induced diabetic rats. The treatment with HTR inhibited the Nox4/TGF-*β*1 signaling pathway and improved the above indicators of oxidative stress.

In addition to oxidative stress, inflammation is also critical to the progression of DN. Clinical studies have shown that inflammatory molecules are independent risk factors, which can predict the development of urinary protein and the incidence of renal failure in diabetic patients [35]. Meanwhile, a binding site of NF*κ*B was found in the promoter region of TGF-*β*1 gene, confirming that the activation of NF*κ*B can induce increased expression of TGF-*β*1 [28, 36]. Apart from this, once the NF*κ*B pathway is activated, p65 transfers from the cytoplasm to the nucleus to upregulate the expression of MCP-1 and proinflammatory cytokines, including IL-1*β* and TNF-*α* [37, 38]. Among them, MCP-1 was found to be significantly correlated with urinary albumin excretion rate [39]. And IL-1 has been demonstrated to increase the permeability of the vascular endothelium and take large part in the proliferation of mesangial cells and matrix synthesis [40]. The expression of TNF in urine and kidney tissues of STZ-induced diabetic rats has been reported to be significantly increased, and inhibition of TNF significantly reduces urine protein excretion [41]. This study showed that the nuclear translocation of p65 was inhibited by HTR treatment. Moreover, the plasma levels and mRNA expression in kidneys of MCP-1, IL-1*β*, and TNF-*α* were all suppressed. Considering the results of oxidative stress and inflammation-related parameters together, the antioxidant and anti-inflammatory effects of HTR are confirmed in DN. In order to better elucidate the target of HTR, molecules, associated with oxidative stress and inflammation-related pathway, were further analyzed.

RETRACTED

AMPK, a serine/threonine kinase, is regulated by the intracellular AMP/ATP ratio [42]. And AMPK is a heterotrimeric protein, composed of catalytic subunit *a* as well as regulatory subunits *β* and *γ*. AMPK activation requires phosphorylation of a critical threonine residue (Thr 172) on *α* subunit. It has been found that the activity of AMPK is inhibited in DN, and AMPK activator can alleviate the proteinuria, mesangial expansion, and increased TGF-*β* levels [15], which are considered to be signs of clinical and pathological changes in DN [43]. The renoprotective effect of AMPK is believed to be related to its antioxidant and anti-inflammatory activities. Studies have identified that AMPK has the ability to reduce Nox4-mediated ROS formation [44]. In addition, AMPK activation has also been reported to reduce inflammation by inhibiting the activation of NF*κ*B [45]. AMPK*α*2 deletion contributes to NF*κ*B translocation to aggravate the inflammatory response in endothelial cells [46].

The body has an antioxidant defense system to resist and repair oxidative damage. The Nrf2/ARE system is now considered one of the most important cellular defense mechanisms against oxidative stress [47]. Under homeostatic conditions, Nrf2, anchored in the cytoplasm, is ubiquitinated and continuously degraded [48]. When the body encounters stresses, Nrf2 is released into the nucleus, binding to the ARE sequence of the downstream target genes to promote the expression of phase II detoxification enzymes, including NQO1 and HO-1, which can alleviate mitochondrial dysfunction and resist excessive oxidative stress [49]. Furthermore, inhibition of Nrf2 can not only result in TLR4/NF*κ*B-mediated proinflammatory response [50], but also promote fibrosis via the activation of TGF-*β*1/Smad pathway [51].

Emerging crosstalk has been found between Nrf2 and AMPK [19]. AMPK can facilitate the nuclear accumulation of Nrf2 by directly phosphorylating it at serine 550 [52]. It can also reduce Nrf2 degradation and increase its activity by inhibiting proteasome activity [53]. It has been reported that AMPK/Nrf2 signaling pathway plays a critical role against oxidative stress and proinflammatory responses to reverse metabolic disorders in DN [54] and nonalcoholic fatty liver disease [31]. Similar findings have also been observed in other diseases. For example, AMPK mediates the amplified activation of Nrf2 signaling to inhibit the lung inflammatory response caused by smoking and ultimately improve chronic obstructive pulmonary disease [55]. In addition, activation of AMPK/Nrf2 signaling pathway can also inhibit neuroinflammation in neurodegenerative diseases [56]. Our study proved that the AMPK/Nrf2 pathway was suppressed in STZ-induced diabetic rats. HTR treatment increased AMPK phosphorylation and promoted the nuclear translocation of Nrf2, thereby upregulating the expression of HO-1 mRNA and protein, although not influencing the NQO1 expression. These results demonstrated that HTR could reverse AMPK/Nrf2 pathway activity in the kidney of STZ-induced diabetic rats.

RETRACTED

In summary, HTR has antioxidant and anti-inflammatory effects. Therefore, it can alleviate renal fibrosis of diabetic rats. And activation of AMPK/Nrf2 pathway may be one of its underlying mechanisms. The findings of this study are summarized in Figure 8.

## 5. Conclusions

HTR has been widely used for the clinical treatment of DN in China. In conclusion, the present study revealed that HTR for removing blood stasis and dredging collaterals inhibited the oxidative stress and inflammation in the kidneys of STZ-induced diabetic rats, thereby reducing proteinuria, protecting renal function, regulating lipid metabolism, improving renal injury, and delaying the progression of fibrosis in DN. Activation of AMPK/Nrf2 pathway may be one of its underlying mechanisms. Therefore, these discoveries suggest that HTR can act as a potential and beneficial compound of TCM for the prevention and treatment of renal fibrosis in DN.

## Figures and Tables

**Figure 1:** Effects of HTR on (a) 24h UTP, (b) Scr, and (c) BUN. Data are presented as mean ± SD (*n* = 7). ^*∗*^*P* < 0.05, ^*∗∗*^*P* < 0.01 vs. control; ^#^*P* < 0.05, ^##^*P* < 0.01 vs. DN.

**Figure 2:** Effects of HTR on (a) RBG and (b) blood lipids. Data are presented as mean ± SD (*n* = 7). ^*∗*^*P* < 0.05, ^*∗∗*^*P* < 0.01 vs. control; ^#^*P* < 0.05, ^##^*P* < 0.01 vs. DN.

**Figure 3:** Effects of HTR on the renal pathology of STZ-induced diabetic rats. HE, PAS, and Masson's trichrome-stained, magnification×400.

**Figure 4:** Effects of HTR on the parameters of oxidative stress in urine and kidneys. (a) SOD activity in kidney cortex detected by colorimetric method. (b) MDA content in kidney cortex detected by colorimetric method. (c) 8-OHdG level in urine detected by ELISA. (d) The immunohistochemical stain of 8-OHdG in kidney cortex (×400). Data are presented as mean ± SD (*n* = 7). ^*∗*^*P* < 0.05, ^*∗∗*^*P* < 0.01 vs. control; ^#^*P* < 0.05, ^##^*P* < 0.01 vs. DN.

RETRACTED

**Figure 5:** Effects of HTR on the parameters of inflammation in serum and kidneys. (a) The levels of TNF*α*, IL-1*β*, and MCP1 in serum detected by ELISA (*n* = 7). (b) The mRNA expression of TNF*α*, IL-1*β*, and MCP1 in serum detected by qRT-PCR. (c) Total and nuclear NF*κ*B expression of rats in kidney cortex measured by western Blot. (d) Quantitative analyses of total NF*κ*B/*β*-actin and nuclear NF*κ*B/H3. Data were presented as mean ± SD (*n* = 3). ^*∗*^*P* < 0.05, ^*∗∗*^*P* < 0.01 vs. control; ^#^*P* < 0.05, ^##^*P* < 0.01 vs. DN.

**Figure 6:** Effects of HTR on Nox4/TGF-*β*1 signaling pathway and the ECM proteins. (a) Representative western blot is shown for Nox4, TGF-*β*1, and *β*-actin. Quantitative analyses are shown for (b) Nox4/*β*-actin and (c) TGF-*β*1/*β*-actin. (d) The immunohistochemical stain of FN and Col IV in kidney cortex (×400). Data were presented as mean ± SD (*n* = 3). ^*∗*^*P* < 0.05, ^*∗∗*^*P* < 0.01 vs. control; ^#^*P* < 0.05, ^##^*P* < 0.01 vs. DN.

**Figure 7:** Effects of HTR on AMPK/Nrf2 signaling pathway. (a) Representative western blot is shown for total AMPK, pAMPK, total Nrf2, nuclear Nrf2, HO-1, NQO1, *β*-actin, and histone H3. Quantitative analyses are shown for (b) pAMPK/total AMPK, (c) total Nrf2/*β*-actin, (d) nuclear Nrf2/H3, (e) HO-1/*β*-actin, and (f) NQO1/*β*-actin. (g) The mRNA relative expression of HO-1 in serum detected by qRT-PCR. (h) The mRNA relative expression of NQO1 in serum detected by qRT-PCR. (i) The protein expression detected by immunofluorescence. Data were presented as mean ± SD (*n* = 3). ^*∗*^*P* < 0.05, ^*∗∗*^*P* < 0.01 vs. control; ^#^*P* < 0.05, ^##^*P* < 0.01 vs. DN.

**Figure 8:** Schematic overview of HTR's effect on renal fibrosis in STZ-induced diabetic rats. ECM accumulation, the characteristic of fibrosis, is a main pathological change in DN. As we all know, oxidative stress and inflammation, which promote each other, are the critical causes of TGF-*β*1-induced excessive synthesis and deposition of ECM in DN. Interestingly, AMPK acts as the upstream of Nrf2. The activation of AMPK/Nrf2 pathway can inhibit the Nox4-induced oxidative stress and attenuate NF*κ*B-induced inflammation. HTR enhances the activity of AMPK/Nrf2 pathway and suppresses oxidative stress and inflammation, thereby decreasing the ECM deposition and delaying the progression of fibrosis in DN (⟶: activated; ⊣: inhibited).

RETRACTED

**Table 1:** Primer sequences for RT-PCR analysis.

Gene	Sequence
IL-1*β*	Fwd: CTCACAGCAGCATCTCGACAAGAG
	Rev: TCCACGGGCAAGACATAGGTAGC

TNF-*α*	Fwd: CCAGGTTCTCTTCAAGGGACAA
	Rev: GGTATGAAATGGCAAATCGGCT

MCP-1	Fwd: GTCACCAAGCTCAAGAGAGAGA
	Rev: GAGTGGATGCATTAGCTTCAGA

HO-1	Fwd: CAGCATGTCCCAGGATTTGTC
	Rev: CCTGACCCTTCTGAAAGTTCCTC

NQO1	Fwd: AGGCTGCTGTGGAGGCTCTG
	Rev: GCTCCCCTGTGATGTCGTTTCTG

GAPDH	Fwd: CTGGAGAAACCTGCCAAGTATG
	Rev: GGTGGAAGAATGGGAGTTGCT

## Data Availability

The datasets used and/or analyzed during the current study are available from the corresponding author on reasonable request.
